The article "Dextran Sulfate Sodium Inhibits Alanine Synthesis in Caco-2 Cells" was retracted in 2012. Reasons: errors in the materials; errors in the methods; errors in the results or conclusions.

# Dextran Sulfate Sodium Inhibits Alanine Synthesis in Caco-2 Cells

**DOI:** 10.3390/ijms12042325

**Published:** 2011-04-04

**Authors:** Zhong Ye, Darya O. Mishchuk, Natasha S. Stephens, Carolyn M. Slupsky

**Affiliations:** 1 Department of Nutrition, University of California, Davis, One Shields Avenue, Davis, CA 95616, USA; E-Mail: zye@ucdavis.edu; 2 Department of Food Science and Technology, University of California, Davis, One Shields Avenue, Davis, CA 95616, USA; E-Mails: domishchuk@ucdavis.edu (D.O.M.); nsstephens@ucdavis.edu (N.S.S.)

**Keywords:** metabolomics, metabonomics, IBD, DSS, NMR, Caco-2, alanine transaminase, Crohn’s disease, ALAT, ALT

## Abstract

To understand and characterize the pathogenic mechanisms of inflammatory bowel disease, dextran sulfate sodium (DSS) has been used to induce acute and chronic colitis in animal models by causing intestinal epithelium damage. The mechanism of action of DSS in producing this outcome is not well understood. In an effort to understand how DSS might impact epithelial cell metabolism, we studied the intestinal epithelial cell line Caco-2 incubated with 1% DSS over 56 hours using ^1^H NMR spectroscopy. We observed no difference in cell viability as compared to control cultures, and an approximately 1.5-fold increase in IL-6 production upon incubation with 1% DSS. The effect on Caco-2 cell metabolism as measured through changes in the concentration of metabolites in the cell supernatant included a three-fold decrease in the concentration of alanine. Given that the concentrations of other amino acids in the cell culture supernatant were not different between treated and control cultures over 56 hours suggest that DSS inhibits alanine synthesis, specifically alanine aminotransferase, without affecting other key metabolic pathways. The importance of alanine aminotransferase in inflammatory bowel disease is discussed.

## 1. Introduction

Crohn’s disease (CD) and ulcerative colitis (UC), both inflammatory bowel diseases (IBD), involve chronic inflammation of the gastrointestinal tract. The etiology and mechanisms of IBD remain unclear, but it is generally agreed to be a complex interplay between the immune system, genetics, and environmental factors. To aid in the understanding of the pathogenesis of the disease, dextran sulfate sodium (DSS) has been used to induce colitis in experimental animal models [1,2]. DSS is a water-soluble polymer of glucose containing up to 20% sulfur with molecular weights ranging from 5,000 to 1.4 million Da. DSS is poorly absorbed after oral administration of enteric coated tablets, and no evidence of systemic absorption has been observed in humans [3]. Depending on the concentration, molecular weight, sulfation, and length of exposure, oral administration of DSS to rodents has been shown to induce acute or chronic colitis that resembles UC [1,4,5]. When supplied with DSS in their drinking water, mice develop colonic mucosal inflammation with ulcerations, body weight loss, and bloody diarrhea that resolves after DSS removal [4]. Chronic inflammation may be induced by administration of a further three to five cycles of DSS [6,7].

The article "Dextran Sulfate Sodium Inhibits Alanine Synthesis in Caco-2 Cells" was retracted in 2012. Reasons: errors in the materials; errors in the methods; errors in the results or conclusions.

Intestinal epithelium damage is a key feature of DSS-induced colitis, characterized by multi-focal areas of mucosal erosion, epithelial cell injury, and significant mucosal infiltration of neutrophils [8]. A recent study involving a mouse model of DSS-induced colitis showed that epithelial apoptosis increased approximately five-fold, mitotic cells decreased by approximately half, and cells with cell cycle arrest at G0 increased two-fold in DSS treated mice as compared to control mice [9].

The effects of DSS have also been studied in cell-culture models. For instance, it has been shown that DSS alters Caco-2 tight junctions, cell cycle metabolism, as well as cytokine release at concentrations ranging from 0.3% to 5% w/v [7,10]. DSS at higher molecular weights and higher concentrations tended to have a greater effect on cell viability [10]. However, it is unclear what metabolic changes happen to colon epithelial cells in the absence of bacteria. In the present study, we apply ^1^H NMR-based metabolomics to study how DSS affects the extracellular metabolites of Caco-2 cells in an effort to understand the mechanism of action of DSS on epithelial cells.

## 2. Results and Discussion

### 2.1. Cell Viability of Caco-2 Cells Treated with DSS Is Similar to Control

To determine whether treated cells were viable after incubation with DSS, a trypan blue dye exclusion assay was performed (Figure 1). At specific time points from 2 to 56 h, numbers of viable cells exposed to 1% DSS were compared to those of controls. No difference in cell viability was found over 56 h. In addition, microscopy did not reveal any significant morphological changes between treated and untreated Caco-2 cells.

### 2.2. Interleukin-6 Level Increases with DSS Incubation

To determine the effect of 1% DSS on expression of interleukin-6 (IL-6), IL-6 assays were performed and compared between control and DSS-treated Caco-2 cells (Figure 2). At all timepoints, the concentration of IL-6 in the cell supernatant was determined to be higher for the DSS-treated cells.

### 2.3. DSS Induces Changes in ^1^H NMR Spectra of Supernatant Derived from Culture of Caco-2 Cells

To determine the effect of 1% DSS on metabolism of Caco-2 cells, ^1^H NMR spectroscopy was performed and compared between control and DSS-treated Caco-2 cell supernatants. Representative spectra from control and 1% DSS-treated cells at 56 h are shown in Figure 3. The concentration of alanine was higher in the control culture in comparison with the DSS-treated culture. Interestingly, no changes in lactate were observed upon incubation with 1% DSS, however, glucose concentrations appeared to be slightly higher in DSS-treated cells, but due to variability between samples, the difference was not significant (Figure 4). Ethanol was a contaminant in all samples, and its concentration was determined to not be significantly different between treated and untreated cells.

The article "Dextran Sulfate Sodium Inhibits Alanine Synthesis in Caco-2 Cells" was retracted in 2012. Reasons: errors in the materials; errors in the methods; errors in the results or conclusions.

Comparison of metabolite concentrations in the cell culture media between the control and DSS-treated Caco-2 cells revealed statistically significant higher concentrations of alanine in the control culture supernatant (Figure 4), with a concentration approximately three times greater than the concentration of alanine in the supernatant of DSS-treated cells. In the media alone, the concentration of alanine is approximately 100 μM. However, in both control and DSS-treated cells the concentration of alanine increases over time to nearly 2 mM for the control, and 600 μM for the DSS-treated cells suggesting that alanine is exported from the cell. Interestingly, the concentration of lactate in the cell culture supernatant was similar between the control and DSS-treated cells. Comparison of metabolites imported into the Caco-2 cells (including glucose, glutamine, and pyruvate) revealed no significant differences between control and DSS-treated cells (Figure 4). Glutamate concentrations were not significantly different between treated and control cells, and α-ketoglutarate was undetectable in the cell culture supernatant.

### 2.4. Discussion

DSS is often used in animal studies to induce colitis [1,2]. However, the metabolic effects of DSS on intestinal epithelial cells have not been characterized to date. In this study, we applied ^1^H NMR spectroscopy to study the effect of DSS on a cell-culture mimic of the human small intestine, Caco-2. Utilizing 1% DSS, we determined that cell viability was unaffected over 56 h, and that a 1.5-fold increase in IL-6 production by Caco-2 cells occurred upon incubation of Caco-2 cells with 1% DSS. This is in agreement to Araki *et al.* [10]. Furthermore, a significant decrease in alanine production was observed when Caco-2 cells were incubated with DSS, but no significant differences were observed in the concentrations of lactate or pyruvate. These observations suggest one of two mechanisms: either the blocking of the alanine transporter, or the inhibition of the enzyme alanine aminotransferase (ALAT) either through blocking of transcription or blocking of the enzyme itself.

The article "Dextran Sulfate Sodium Inhibits Alanine Synthesis in Caco-2 Cells" was retracted in 2012. Reasons: errors in the materials; errors in the methods; errors in the results or conclusions.

Alanine transport in Caco-2 cells occurs via system B, which is a sodium dependent chloride-independent transporter that also transports glutamine [11]. If DSS were blocking this transporter, changes in the transport of glutamine would be expected (Figure 5). However, no significant change in the concentration of glutamine was observed in the cell supernatant of DSS-treated versus control cells. Thus the lower concentration of alanine is unlikely due to the blockage of the alanine transporter. Although system B is a sodium-dependant transporter, it has been previously determined that sodium concentration does not affect maximal alanine influx [12,13]. Even so, the addition of 1% DSS to the cell culture only changed the conductivity by a small amount (16.7 mS/cm *versus* 15.4 mS/cm in the control media).

Alanine aminotranferase (ALAT) is an enzyme that catalyzes the transfer of the α-amino group from glutamate to pyruvate forming alanine and α-ketoglutarate. Inhibition of this enzyme would impact synthesis of alanine, but not necessarily change the concentration of other metabolites or affect other cellular pathways as pyruvate has many fates in the cell including the formation of lactate, other amino acids, and can enter the TCA cycle. α-Ketoglutarate can also enter the TCA cycle. If the reason for decreased alanine in the cell culture media is due to the inhibition of ALAT, it is likely that it occurs either through direct inhibition of the enzyme or through inhibition of transcription. In either case, the enzyme still functions as the concentration of alanine in the medium of DSS-treated cells does increase from the baseline level in the media over 56 hours.

The fact that ALAT is somehow affected by DSS is an interesting finding. In a study involving 123 IBD patients, it was determined that 49/50 CD patients had subnormal serum ALAT levels, whereas only 1/67 patients with UC had subnormal ALAT on one or more occasions [14]. Interestingly, however, in a study of 544 patients, it was determined that ALAT was increased in concentration in the serum, with no specific association to IBD activity [15]. In another study, total enteral nutrition of pediatric patients was shown to be associated with a transient hypertransaminasemia and no other evidence of liver disease [16]. In a study involving IL-10 gene deficient mice, it was determined that in both wild-type and gene-deficient mice, treatment of mice with dinitrobenzene sulfonic acid (DNBS) resulted in a substantial increase in serum ALAT [17]. However serum ALAT did not appear significantly different from control in 5% DSS-treated mice [18]. Of importance, it was determined that the concentration of alanine in the colonic mucosa of patients with both UC and CD was decreased as compared to normals [19]. Moreover, alanine was shown to be significantly higher in fecal samples from CD patients, but not UC patients, as compared to control [20].

The article "Dextran Sulfate Sodium Inhibits Alanine Synthesis in Caco-2 Cells" was retracted in 2012. Reasons: errors in the materials; errors in the methods; errors in the results or conclusions.

Taken together, regulation of ALAT activity, either through direct inhibition of the enzyme or inhibition of transcription, has an association with inflammatory bowel disease, and in particular Crohn’s disease. Whether it is directly related to the pathogenesis of CD, or is a consequence of the disease itself remains to be elucidated. The fact that in human patients serum ALAT deviations from normal may be transient in nature, and in most cases do not appear to be associated with liver disease suggests that there may be a dietary or bacterial flora connection. Although ALAT activity has often been thought of as an indicator of hepatic function, the increase in serum values of ALAT may be related to changes in the intestinal tissue itself, with changes in intestinal metabolism potentially signaling changes in hepatic ALAT expression. Indeed it has been shown that patients with CD have increased insulin secretion [21], and that higher ALAT levels are associated with impaired glucose tolerance [22]. Of significance, it has been shown that p300 and c-Myb regulate ALAT gene transcription, and that insulin levels affect expression of these factors [23] thereby affecting ALAT gene expression. We are currently investigating whether DSS directly inhibits ALAT or inhibits transcription, and whether serum levels of ALAT can affect the action of DSS.

## 3. Experimental Section

### 3.1. Caco-2 Preparation and Reagents

The human Caco-2 cell line has been widely used as an *in vitro* model of the intestinal epithelium [24]. In this study, Caco-2 cells were obtained from American Tissue Culture Collection (ATCC, Manassas, VA, USA) at passage 18 and experiments were performed with cells from passages 25–30. Caco-2 cells were cultured in Dulbecco’s modified Eagle’s minimum essential medium (DMEM, HyClone, Logan, UT, USA) supplemented with 25 mM glucose, 10% fetal bovine serum (FBS), 1% nonessential amino acids, 4 mM L-glutamine and 1% penicillin-streptomycin solution at 37 °C with 5% CO_2_. Dextran sulfate sodium (DSS, MW 36,000–50,000, MP Biomedicals LLC, Solon, OH, USA) was dissolved in culture media and filter-sterilized using a 0.2 μm filter. To test the effect of DSS on Caco-2 cells, cells were seeded onto 24-well plates (Costar, Corning, NY, USA) at a density of 1 × 10^4^ viable cells/cm^2^. After 90–100% confluency, the Caco-2 cell monolayers were allowed to differentiate for an additional 14 days. Fully differentiated cell monolayers were incubated with or without 1% DSS in cell culture media for 2 to 56 h. The Caco-2 cells at different time points after DSS addition were observed under an Olympus IX71 inverted microscope equipped with a digital camera using MetaMorph software. Images of Caco-2 cells were taken at 40X magnification. 1.0 mL aliquots of supernatant samples were collected at different time points, centrifuged at 14,000 rpm for 20 min to remove cellular debris, and stored at −80 °C until further analysis.

The article "Dextran Sulfate Sodium Inhibits Alanine Synthesis in Caco-2 Cells" was retracted in 2012. Reasons: errors in the materials; errors in the methods; errors in the results or conclusions.

### 3.2. Caco-2 Cells Viability Test

Caco-2 cells were incubated with DSS in 24 well plates as described above. At each time point, cells were collected from the wells using 0.5 mL of 0.25% trypsin with 0.2 g/L EDTA (HyClone, Logan, UT, USA) and re-suspended in 1 mL of serum-free medium. The viability of control cells and cells incubated with DSS were determined using a Bright Line hemacytometer (Hausser Scientific, Horsham, PA, USA) and the trypan blue dye exclusion test. Results of viability are expressed as the percentage of the values obtained for control cells. All experiments were performed four times.

### 3.3. IL-6 Assay

Caco-2 cells were incubated in 24-well plates (Costar) and cell culture supernatants were collected as described above. IL-6 assays were performed using human IL-6 ELISA Ready-Set-Go kit (eBioscience, Inc., San Diego, CA, USA) according to manufacturer instructions.

### 3.4. NMR Sample Preparation, Spectroscopy and Analysis

*Sample preparation:* Samples were prepared by thawing the frozen supernatant and filtering though a 3000 MW cutoff filter (Pall Life Sciences, Ann Arbor, MI, USA). 585 μL of filtered sample was mixed with 65 μL of Internal Standard (IS) (5mM DSS-d6 (3-(trimethylsilyl)-1-propanesulfonic acid-d6) with 0.2% NaN3, in 99.8% D_2_O and the pH was adjusted to 6.8 ± 0.1. A 600 μL aliquot of each sample was transferred to a 5-mm NMR tube and stored at 4 °C until NMR data acquisition.

*NMR spectroscopy:* All one-dimensional NMR spectra of the samples were acquired using the first increment of the standard NOESY pulse sequence on a Bruker AVANCE 600 MHz NMR spectrometer equipped with a SampleJet. All spectra were recorded at 25 °C with a 12 ppm sweepwidth, 2.5 s recycle delay, 100-ms τ_mix_, an acquisition time of 2.5 s, 8 dummy scans, and 32 transients. ^1^H saturation of the water resonance was applied during the recycle delay and the 100 ms τ_mix_. All spectra were zero-filled to 128k data points and multiplied by an exponential weighting function corresponding to a line-broadening of 0.5 Hz.

The article "Dextran Sulfate Sodium Inhibits Alanine Synthesis in Caco-2 Cells" was retracted in 2012. Reasons: errors in the materials; errors in the methods; errors in the results or conclusions.

*Spectral analysis:* Analysis of the NMR data was accomplished through targeted profiling using the Chenomx NMRSuite v6.1 (Chenomx Inc., Edmonton, Canada) [25]. A total of 39 metabolites were identified and quantified representing 99% of the spectral area.

### 3.5. Statistical Analysis

All data, including the concentrations derived from the ^1^H NMR spectra, IL-6 ELISA results, and viability of Caco-2 cells, are presented as mean ± SD. The difference in levels of variable between treatment and control were evaluated for individual values using the Student’s t-test. *P-*values of <0.05 were considered to be statistically significant.

## 4. Conclusions

The goal of this study was to understand the effect of DSS on Caco-2 cell metabolism. Although cell viability was similar, and IL-6 production was increased approximately 1.5 times, the only major metabolite difference observed when Caco-2 cells were incubated with 1% DSS was a decrease in alanine concentration in the cell culture medium as compared with controls. Since the concentration of glutamine and other amino acids were unaffected, we ruled out the possibility that DSS inhibited alanine transport across the membrane. These results suggest that either transcription of alanine aminotransferase is inhibited, or the enzyme itself is inhibited. This study emphasizes that alanine aminotransferase has a direct relationship with inflammatory bowel disease, and in particular CD, and may provide a more thorough understanding of the pathogenesis of CD in addition to the metabolic mechanisms for DSS-induced colitis in animal models. Work is currently under way to determine how alanine aminotransferase is inhibited by DSS.

## Figures and Tables

**Figure 1.** Incubation of Caco-2 with dextran sulfate sodium (DSS) does not affect viability or morphological characteristics of Caco-2. **(A)** Numbers of viable cells were determined using the trypan blue dye exclusion method. Percent viability was expressed as the percentage of growth compared to total cells at each time point; **(B)** Images of Caco-2 cells using microscopy at 40× were acquired using an Olympus digital camera. Each time point for both treated and untreated groups represents the mean of four determinations.

**Figure 2.** Secretion of IL-6 in cell culture medium by control (□) and 1% DSS-treated ( ) Caco-2 cells. Supernatants were collected for each of control and DSS-treated cells at 2, 6, 8, 10, 24, 32, and 56 hours, and IL-6 levels were measured, and averaged. Results therefore represent the mean of 28 determinations ± SD, *p* = 0.00003.

**Figure 3.** Representative 600 MHz ^1^H NMR spectra obtained from cell supernatant extracts from control and DSS-treated Caco-2 cells. IS (internal standard) represents sodium 2, 2-dimethyl-2-silapentane-5-sulfonate used as chemical shift reference. Ethanol is a contaminant.

The article "Dextran Sulfate Sodium Inhibits Alanine Synthesis in Caco-2 Cells" was retracted in 2012. Reasons: errors in the materials; errors in the methods; errors in the results or conclusions.

**Figure 4.** Comparison of the concentration of metabolites in control (□), and 1% DSS-treated ( ) Caco-2 cell culture supernatants. All metabolites in cell culture supernatants were collected for each of control and DSS-treated cells at 10, 24, 32, and 56 hours, and metabolites were measured, and averaged. Results therefore represent the mean of 16 determinations ± SD, and * *p* < 0.00001.

**Figure 5.** Schematic of alanine metabolism in Caco-2 cells. Here it is shown that Caco-2 cells absorb glucose, glutamine, and pyruvate from the medium and produce lactate and alanine that are released. Over time, glucose, glutamine, and pyruvate concentrations decrease in the medium while lactate and alanine concentrations increase.
